RETRACTED

# Strengthening public health surveillance through blockchain technology

**DOI:** 10.3934/publichealth.2019.3.326

**Published:** 2019-09-02

**Authors:** Sudip Bhattacharya, Amarjeet Singh, Md Mahbub Hossain

**Affiliations:** 1 Department of Community Medicine, Himalayan Institute of Medical Sciences, Dehradun, India; 2 Department of Community Medicine, School of Public Health, Postgraduate Institute of Medical Education and Research, Chandigarh, India; 3 Department of Health Promotion and Community Health Sciences, School of Public Health, Texas A & M University, Texas, USA

**Keywords:** blockchain technology, telemedicine, medical informatics, disease outbreaks, population surveillance

## Abstract

Blockchain technology is a decentralized system of recording data and performing transactions which is increasingly being used across many industries, including healthcare. It has several unique features like the validation of transaction processes, prevention of systems failure from any single point of transaction, and approval of data sharing with optimal security, to name a few. At the hospital level, blockchain technologies are used in the electronic medical records systems, insurance claims, billing management, and so on. Moreover, this technology is helpful to manage logistic and human resources to achieve the quality of care in learning health systems. In many countries, blockchain is being used to promote patient-centered care by sharing patient data for remote monitoring and management. Furthermore, blockchain technology has the potential to strengthen disease surveillance systems in cases of disease outbreaks resulting in local and global health emergencies. In such conditions, blockchain can be used to identify health security concerns, analyze preventive measures, and facilitate decision-making processes to act rapidly and effectively. Despite its limitations, research, and practice based on blockchain technology have shown promises to strengthen health systems around the world with a potential to reduce the global burden of diseases, mortality, morbidity, and economic costs.

## 1. Introduction

In the twenty-first century, many scientific innovations have changed the means of day-to-day communication, transactions, and decision-making. Blockchain is such a technology, which is being considered as one of the most significant inventions since the discovery of internet [1]. It is also popularly termed as the next generation of “internet of things” [2]. The rise of Bitcoin and other cryptocurrencies have certainly helped blockchain to get the spotlight across the globe. However, the experts believe that blockchain is more than cryptocurrencies and that it may offer greater benefits to the users of complex systems [1],[3]. Blockchain technology is commonly used for online money transfers, bank payments. It is also used in automobile industries, cybersecurity, exit polls, education sector, insurance companies, and forecasting time trends [4]. Recently, blockchain technology has gained popularity among several domains, including health systems. This is because it offers a safer and decentralized database that can operate independent of a centralized administrator [3]. According to Angraal et al., unique selling proposition of the blockchain system is that, once digital validation takes place, the network itself streamlines and validates the subsequent process of transaction. It safeguards the transaction history, and allows data to be transferred directly between third parties [5]. In this article, we discuss how blockchain technology works and how it can be used in complex situations like strengthening public health surveillance.

RETRACTED

## 2. Blockchain and its applications

A blockchain is defined as “A distributed system (decentralized) which performs the dual function of recording and storing the records of the transaction. In this blockchain, the data is located in a network of personal computers called ‘nodes’ without any central control.” (Figure 1).

**Figure 1.** Centralized (a) and decentralized network (b).

The main advantage of this decentralized technology is that all the dealings or variations in the data are captured in with real-time updates across the network [6]. So, the information gets stored in each node is similar, it is permanent. It can't be distorted. Hence this technology is transparent and autonomous. Also it improves the quality of shared data between different stakeholders [7]. In this system, to validate the transaction, cryptographic algorithms are used [8]. This is different from “trust-in-the-third-party” mechanism, where an online transaction takes when for two willing parties approve the transaction by a digital signature [2]. Moreover, blockchain overcomes the challenge of “single point failure” which is common in centralized information management systems [9]. Basically, in routine used so far, the centralized healthcare systems lack the advantages offered by blockchain including transparency and trust, data security and privacy, cost-effectiveness, verifiability of data, fast and real-time data transfer to the all trusted parties [10].

## 3. Types and uses of blockchain

There are two main types of blockchains:

(1). Open access blockchains-Where all records are visible to the stakeholders

(2). Limited access blockchains-Where the access of data/information is restricted [11]. Open access blockchains are more appropriate to the health sector. Till date, bitcoin (most popular applications of block chain technology) uses this technology for cryptocurrency [12].

RETRACTED

## 4. Blockchain technology in healthcare

(a). *At hospital level:* Blockchain is one of the popular technologies used in electronic medical records (EMR) in modern hospital ecosystems in the industrialized nations. Several features including decentralization, data provenance, and robustness have made blockchain technology suitable for storing, managing, and sharing protected health information in EMR [13]. For example, health chain is a blockchain-based EMR system which used hyperledger fabric by IBM [14]. This technology helps to achieve scalable data security and optimize the performance of the EMR system. Arguably, blockchain is considered to improve transactions in billing section, insurance claims, and surveillance measures like nosocomial infection surveillance [14]. The advantage of this technology is that a lot of data can be stored, processed and shared with the stakeholders, very swiftly, without any link failure/delay [16]. According to Peterson et al., it can reform health database interoperability with in-built authentication controls, which lowers the risk of data theft [12].

(b). *Resource management in health systems:* Blockchain can facilitate managing logistic and human resources in healthcare systems. For example, counterfeit medications and instruments below standard can be supplied to healthcare systems from external vendors. Use of blockchain can validate the quality standards at different nodes of supply chain management and inform the respective authorities about suspected discrepancies [17]. Moreover, human resource management in the digital age requires storing and using employee data for attendance, leaves, performance appraisal, and security measures with complex authentication processes. Use of blockchain can make such processes efficient and contribute to the development of smarter health services organizations.

(c). *Patient-level applications:* Due to its decentralized features protecting data safety concerns, blockchain is increasingly being used to share the health data with patients and their caregivers. Such patient empowerment initiatives are also fostering meaningful use of health information technology and improving patient-provider communication in the digital platforms [18]. Furthermore, blockchain-based mHealth interventions are enabling remote patient monitoring through use of biosensors, thus bridging the access gaps in patient-level health services [19].

(d). *Disease Surveillance at community level:* Surveillance is defined as “systematic, ongoing collection, collation, and analysis of data and the timely dissemination of information to those who need to know so that the action can be taken [20]”. It is done for both communicable diseases and noncommunicable diseases by all the national health systems according to the national priorities as per WHO's International Health Regulations (IHR). For example, deadly virus like Nipah can travel across the globe within 36 hours and can cause pandemic by compromising health security due to rapid and uncontrolled urbanization and globalization [21]. Communicable disease surveillance is an ongoing, complex and inefficient process, because a huge number of self-regulating organizations report to a centralized information system. So, it is a challenging task to keep the information flow seamlessly in a timely manner [15],[22]. Moreover, there is no incentives are allotted for the routine staffs. The sequence of events after the reporting of a case by a health worker until the timely action is depicted in Figure 2.

RETRACTED

**Figure 2.** Sequence of events in disease surveillance system.

Blockchain could help these independent organizations to manage data more efficiently during the pandemics [23]. It could also help track information for ongoing public health emergencies, like road traffic accidents, illicit drug use, opioid misuse, and so on [24]. When the block chain technology is used in a public health domain, these networks might be able to automate secure data sharing and storage at different levels of healthcare organizations.

This technology has a potential to give real time data/information by sensing potential outbreaks or bioterrorism. Hence, if vaccinations, antibiotics, and other disease control measures are instituted promptly, massive casualties can be prevented. For example, fake news on social media against vaccination have critically impacted public health in recent years [25]. Huckle et al. reported a blockchain based approach to identify the origins of such harmful contents and identify the population at risk in digital communication [26]. This highlights the potential of blockchain to improve public health surveillance in the era of digitalization.

Nowadays, most of the countries use machine learning techniques in surveillance. There are certain unique and added advantages of blockchain technology over machine learning techniques. The blockchain predominantly blocks malicious activities, like data hacking and duplication [27]. Additionally, the combination of blockchain technology with Artificial Intelligence (AI) is like addition of “cherry on the cake” to medical research and health sector [28].

RETRACTED

There is also tremendous scope for integration with geographical information system (GIS) to expedite the routine epidemic investigations, drug and vaccine supply chain management. The other critical aspect is that by ensuring transparency and correct reporting, as in the case of reporting deaths from the particular outbreak, the blockchain overcomes the limitations of already-present in the district health information systems. The following schematic illustration (Figure 3) shows how the blockchain application in surveillance systems enhances the activities for ensuring health security.

**Figure 3.** Application of block chain in surveillance system.

Under these three broad categories of disease control action points namely prevent, detect and respond as shown in Figure 3, there is a great scope for real-time surveillance for detection of Non-Communicable Diseases (NCD). This also comes under the Global Health Security Agenda (GHSA) action packages.

By applying real-time surveillance, early risk factors detection for NCDs can be ensured. In addition, by capacity building of medical and health staff, the emergency response can be overcome through effective supply chain systems [29]. The summary of the NCD activities and GHSA action package activities are shown in Table 1.

**Table 1.** Real time surveillance for NCDs within the global health security agenda.

GHSA category	GHSA action package	NCD RELATED activity
Detect	Real time surveillance	1. Strengthen cancer registries
		2. Support tobacco use surveillance
		3. Birth defects surveillance due to zika virus
		4. Include NCD indicators in current surveillance systems
		5. Support inclusion of Electronic Medical Records
		6. Implement for health data

## 5. Limitations

Blockchain technology has several limitations which include use of the technology without adequate security and privacy measures, lack of frameworks for implementation and regulation, concerns for cost-effectiveness and interoperability [30]. These challenges can be overcome by gradual scalability and upgradeability.

## 6. Discussions and conclusions

The case of Taiwan is an excellent example of the application of this revolutionary blockchain technology [31]. In Estonia, the complete public health infrastructure is being operated using blockchain [32]. Other examples include countries such as the UK, USA, and Canada, where such real-time surveillance systems have been implemented in many of their departments. In England, at the national level, they have implemented it in their Emergency Department Syndromic Surveillance System. Emergency Department Syndromic Surveillance has been implemented by Canada at the regional level. Another excellent example of this application is the European Antimicrobial Resistance Surveillance Network [23],[33]. Hence, we may conclude that, blockchain applications can retain the prime characteristics of ideal disease surveillance. It can be more effective and prompter than the traditional surveillance in terms of coverage, durability, consensus, selective privacy, uniqueness and timing. Blockchain technology holds great promise in overpopulated and low-income countries like India, Pakistan, Africa (where the health systems are prone to epidemic and pandemic) by strengthening the capacity of the countries with simplified early warning surveillance for diseases of epidemic potential by reducing the mortality, morbidity and economic costs. It is high time to incorporate blockchain technology for the low-income countries within the existing surveillance systems for health system strengthening.
